# Application of Visual Artificial Airway in Patients with ARDS Assisted by Pulmonary Ultrasound

This article has been retracted.

**DOI:** 10.1155/2022/2719016

**Published:** 2022-08-12

**Authors:** Liuqin Xia, Jianping Ma, Lingli Hu, Ying Zhu, Mengyuan Diao

**Affiliations:** Department of Intensive Care Unit, Affiliated Hangzhou First People's Hospital, Zhejiang University School of Medicine, Hangzhou, Zhejiang, China

## Abstract

**Objective:**

To explore the application of pulmonary ultrasound in visual nursing of artificial airway in patients with acute respiratory distress syndrome (ARDS).

**Methods:**

Seventy-eight ARDS patients with mechanical ventilation admitted from February 2021 to January 2022 were included and divided into the intervention group and the control group. The control group was given routine airway nursing, and the intervention group was given visual airway nursing management through lung ultrasound. The arterial blood gas analysis indexes, mechanical ventilation time, ICU treatment time, total hospitalization time, aspiration, and the incidence of ventilator-associated pneumonia (VAP) were compared between the two groups.

**Results:**

After treatment, PaO_2_, PaCO_2_, SPO_2_, and oxygenation indexes were significantly improved compared with those before treatment, and the indexes in the intervention group were better than those in the control group after treatment, and the differences were statistically significant (*P* < 0.05). The mechanical ventilation time (5.39 ± 0.68 vs. 7.92 ± 0.59 days), ICU treatment time (8.05 ± 1.14 vs. 10.71 ± 1.16 days), and total hospitalization time (12.05 ± 2.20 vs. 15.68 ± 2.18 days) in the intervention group were significantly shorter than those in the control group (*P* < 0.05). The incidences of aspiration (2.56% vs. 15.38%) and VAP (5.13% vs. 20.51%) in the intervention group was significantly lower than that in the control group (*P* < 0.05).

**Conclusion:**

The application of visual artificial airway management assisted by lung ultrasound in ARDS patients can shorten the treatment time and hospitalization time of mechanical ventilation, reduce the incidence of aspiration and VAP, and improve the prognosis of patients.

## 1. Introduction

Acute respiratory distress syndrome (ARDS) is an acute inflammatory injury disease of the lungs [1]. Recent studies have found that 23% of patients receiving mechanical ventilation in intensive care units have ARDS, and the mortality rate can reach 40% [2]. The high mortality rate is caused by the severity of lung injury [3]. With the advances of ultrasound technology, pulmonary ultrasound is known as a visual “stethoscope” [4, 5]. The characteristics of real-time, safe, repeatable, visualized, and radiation-free of pulmonary ultrasound are irreplaceable advantages of X-ray and CT, which have been widely used in patients with severe condition assessment and monitoring [6, 7]. However, there are few studies on artificial airway care for severe patients, and the quality of artificial airway care for ARDS patients will directly affect the control of pulmonary infection and improvement of ventilation and blood flow. High-quality airway management can reduce pulmonary complications, shorten hospital stay, and reduce patient mortality [8]. The purpose of this paper is to carry out individualized care management of artificial airway in ARDS patients with the help of “visualization” of pulmonary ultrasound.

The pulmonary ultrasound is a tool used in emergency departments and intensive care units for rapid diagnosis and monitoring of treatment. Transthoracic lung ultrasound has high sensitivity, specificity, and diagnostic accuracy in the diagnosis of pneumonia, pneumothorax, pulmonary embolism, pleural effusion, and interstitial pulmonary syndrome. The pulmonary ultrasound can provide visual image basis for postural drainage, chest percussion, abdominal breathing training, and other operations, so as to carry out dynamic effect evaluation, so that patients' airway secretions can be effectively drained, and improve their ventilation and blood flow. On the other hand, it can help patients with ARDS to train diaphragm function and promote their early recovery.

## 2. Patients and Methods

### 2.1. Population

The present study was designed as a prospective study. We included the patients according to the following inclusion and exclusion criteria from the beginning of 2021. A total of seventy-eight patients with ARDS who received mechanical ventilation from February 2021 to January 2022 were selected as the study subjects. The inclusion criteria were as follows: (1) ARDS patients receiving artificial airway and mechanical ventilation duration of more than 3 days; (2) only adult patients were included; (3) acute physiology and chronic health evaluation II (APACHE II) ≥ 15 [9]; and (4) informed consent signed by family members and volunteered to participate in the study. The exclusion criteria were as follows: (1) positive sputum culture before the establishment of artificial airway; (2) patients died during mechanical ventilation or family members giving up treatment; and (3) pregnant patients and patients' age younger than 18 years old were excluded. The subjects were randomly divided into the intervention group and the control group (39 cases in each group), and there was no difference in basic condition between the two groups (*P* > 0.05, Table 1).

### 2.2. Interventions

#### 2.2.1. Control Group

The control group was given routine artificial airway care [10]: (1) if the condition permits, the patient's head of bed should be raised 30-45° and should be turned over every 2-3 h; (2) balloon pressure is maintained at 25-30 cmH_2_O; (3) sputum drainage was promoted by airway heating and humidification, atomization, and inhalation; (4) lung buttoning, vibration expectoration, and airway suction should be carried out as required; (5) intermittent subglottic attraction to prevent aspiration; and (6) use 2% chlorhexidine for oral wiping, brushing teeth, or rinsing every 4-6 h.

#### 2.2.2. Intervention Group

In addition to conventional artificial airway care measures, the intervention group underwent “visual” management: (1) a visual airway management team was established, including a head nurse, ultrasound qualified doctors (*n* = 2), respiratory therapists (*n* = 3), a deputy chief nurse (*n* = 2), a chief nurse (*n* = 4), and a nurse (*n* = 6); (2) after the patient was admitted to the ICU, ultrasound-qualified doctors evaluated the patient on the basis of X-ray examination and determined the patient's pulmonary infection, atelectasis, pulmonary edema, and exudation [11]. Based on the evaluation results, the best positions such as semidecubitus, healthy side decubitus, affected side decubitus, low head and high feet, and prone position were prescribed; (3) when nurses turn over patients, the implementation of the best position of the lungs after targeted lung button back, vibration expectoration, atomization inhalation, and other nursing measures to promote effective sputum drainage (change the position before and after the airway suction), if necessary to the patients with atelectasis lung drum treatment; (4) during postural drainage, enteral nutrition was suspended, and patients' vital signs were closely monitored; and (5) ultrasound-qualified doctors performed dynamic assessment of pulmonary ultrasound and diaphragmatic function assessment on a daily basis to determine whether patients could be trained for early pulmonary respiratory function [12].

### 2.3. Outcomes

The arterial blood gas index, mechanical ventilation time, ICU treatment time, total hospitalization time, and incidence of aspiration and VAP were compared between the two groups before and after treatment.

### 2.4. Statistical Analysis

Statistical software SPSS (version 18.0) was used for statistical analysis. The measurement data of the normal distribution were expressed as mean ± standard deviation (mean ± sd), and the *t*-test was used to compare the measurement data between the two groups. The data of nonnormal distribution were expressed as median and quartile (25% quartile to 75% quartile), and the measurement data between the two groups were compared using a nonparametric test. The chi-square test was used to compare the rates between the two groups. *P* < 0.05 indicated that the difference was statistically significant.

## 3. Results

### 3.1. Comparison of Arterial Blood Gas Analysis between the Two Groups

A total of 78 patients were included, 39 patients in the intervention group and 39 patients in the control group. After treatment, PaO_2_, PaCO_2_, SPO_2_, and oxygenation indexes were significantly improved, and all indexes in the intervention group were better than those in the control group, the differences were statistically significant (*P* < 0.05, Table 2).

### 3.2. Comparison of Mechanical Ventilation Time, ICU Treatment Time, and Total Hospitalization Time between the Two Groups

The mechanical ventilation time, ICU treatment time, and total hospitalization time in the intervention group were significantly shorter than those in the control group (*P* < 0.05, Table 3).

### 3.3. Comparison of the Incidence of Aspiration and Ventilator-Associated Pneumonia between the Two Groups

The incidence of aspiration and ventilator-associated pneumonia in the intervention group was 2.56% and 5.13%, respectively, significantly lower than 15.38% and 20.51% in the control group (*P* < 0.05, Table 4).

## 4. Discussion

The only effective treatment for ARDS patients is mechanical ventilation [13, 14]. Correct mechanical ventilation treatment can significantly reduce the mortality of patients; otherwise, it will further increase the patient's condition, resulting in ventilator-related lung injury (VILI) [15, 16], or even endanger the patient's life. Mechanical ventilation treatment needs to be established on the basis of an effective artificial airway, which is prone to balloon leakage, accumulation of airway secretions, accumulation of condensation water in respiratory pipes, aspiration, and VAP occurrence. The quality and safety of care of artificial airway directly affect the effect of mechanical ventilation [17, 18]. At present, there is no unified standard for the artificial airway care in clinical practice, and most care interventions are carried out through the prevention of complications [19].

As a pulmonary diagnostic tool, pulmonary ultrasound can be traced back to the 1960s [20], but it is a relatively new research field in the study of ARDS, mainly applied to the monitoring of pulmonary edema [21]. The international consensus conference on pulmonary ultrasound promoted by the World Alliance for Critical Care Ultrasound standardized the naming and technology of pulmonary ultrasound and provided recommendations for its use in clinical practice, making it play an increasingly important role in bedside chest imaging, fluid resuscitation, and pneumothorax and pleural effusion diagnosis in ARDS patients [15–17, 22–24]. However, there are few studies on artificial airway care. In the present study, the medical staff assisted to implement targeted and individualized care interventions by establishing a pulmonary ultrasound visual airway management team. Using ultrasound results, the nursing staff performed drainage of the lung in the optimal position, such as the left lung infection patients with heavier, to line right side position and strengthen the left lung buckle back, the vibration row phlegm, and according to the lungs under ultrasonic diaphragm function assessment, implementation of respiratory function training, in the process of training the patient by deep breathing slowly, breathing skills, and the ability to increase the oxygen diffusion, increase alveolar ventilation [8] (Figure 1).

In this study, the visualization of pulmonary ultrasound was applied to the artificial airway nursing of ARDS patients, and the results are as follows: (1) after treatment, the arterial blood gas analysis such as PaO_2_, PaCO_2_, SPO_2_, and oxygenation indexes in the intervention group were significantly improved compared with those in the control group, and the differences were statistically significant (*P* < 0.05, Table 2), which may be related to effective ventilation and drainage in the best position assessed by ultrasound; (2) compared with the control group, mechanical ventilation time (5.39 ± 0.68 vs. 7.92 ± 0.59), ICU treatment time (8.05 ± 1.14 vs. 10.71 ± 1.16), total hospitalization time (12.05 ± 2.20 vs. 15.68 ± 2.18) in the intervention group were significantly shortened (*P* < 0.05, Table 3); (3) the incidence of aspiration (2.56%) and VAP (5.13%) in the intervention group was significantly lower than that in the control group (15.38% and 20.51%) (*P* < 0.05, Table 4), which may be related to timely care intervention after dynamic ultrasound evaluation, as well as significantly shorter mechanical ventilation time and hospital stay.

However, this study also has some limitations. First of all, we only used the data from a single center. Second, the sample size was relatively small, that the selection bias might be not avoided. Third, this study only focused on the period of ICU hospitalization; we lack data on follow-up on long-term prognosis.

In conclusion, the application of pulmonary ultrasound in artificial airway care for ARDS patients can effectively improve the effective ventilation of patients; shorten the treatment time of mechanical ventilation, ICU treatment, and hospital stay; reduce the incidence of aspiration and VAP; and improve the prognosis of patients.

## Figures and Tables

**Figure 1:** Ultrasound contrast of lungs before and after prone position ventilation.

**Table 1:** Comparison of basic conditions between the two groups (mean ± sd)/[*n*(%)].

Groups	*N*	Gender		Age (years)	APACHE II score
		Male	Female		
Control group	39	26 (66.67)	13 (33.33)	43.18 ± 12.65	25.67 ± 4.81
Intervention group	39	25 (64.10)	14 (35.90)	43.57 ± 12.48	25.39 ± 5.08
*P*		0.812		0.672	0.772

**Table 2:** Comparison of arterial blood gas analysis between the two groups (mean ± sd, *n* = 39).

Groups	PaO_2_ (mmHg)	PaCO_2_ (mmHg)	SPO_2_ (%)	Oxygenation index (mmHg)
Control group				
Prior to treatment	50.61 ± 6.12	67.32 ± 8.49	89.29 ± 1.48	183.45 ± 13.04
Posttreatment	63.54 ± 7.56^①^	49.47 ± 5.24^①^	91.35 ± 2.01^①^	217.21 ± 20.48^①^
Intervention group				
Prior to treatment	50.76 ± 6.03	67.09 ± 8.72	89.36 ± 1.45	183.96 ± 13.12
Posttreatment	71.92 ± 7.84^①②^	44.18 ± 5.06^①②^	93.47 ± 2.13^①②^	245.08 ± 24.75^①②^

Note: compared with before treatment, ^①^*P* < 0.05; compared with the control group, ^②^*P* < 0.05.

**Table 3:** Comparison of mechanical ventilation time, ICU treatment time, and total hospitalization time between the two groups (mean ± sd).

Groups	*n*	Mechanical ventilation time	ICU treatment time	Total hospitalization time
Intervention group	39	5.39 ± 0.68	8.05 ± 1.14	12.05 ± 2.20
Control group	39	7.92 ± 0.59	10.71 ± 1.16	15.68 ± 2.18
*P*		0. 001	0. 005	0. 018

**Table 4:** Comparison of the incidence of aspiration and ventilator-associated pneumonia (VAP) between the two groups.

Groups	*n*	Aspiration (%)	Ventilator-associated pneumonia (%)
Intervention group	39	1 (2.56)	2 (5.13)
Control group	39	6 (15. 38)	8 (20. 51)
*P*		0. 033	0. 032

## Data Availability

Data is available on request from the authors.
